# Cleft Lip and Palate Associated With the Phonetic Function: A Systematic Review

**DOI:** 10.7759/cureus.104316

**Published:** 2026-02-26

**Authors:** Anahí Montesdeoca, Dennys Tenelanda Lopez, Mauro Costales, Alejandro Pallo, Sandra Quisiguina

**Affiliations:** 1 Dentristy, Ministry of Public Health, Ambato, ECU; 2 School of Dentistry, National University of Chimborazo, Riobamba, ECU; 3 School of Nutrition and Dietetics, Higher Polytechnic School of Chimborazo, Riobamba, ECU

**Keywords:** cleft lip, cleft palate, nasality, phonemes, phonetic function

## Abstract

Cleft lip and palate (CLP) are congenital malformations of the craniofacial complex that disrupt the structure and function of the stomatognathic system, particularly articulation and phonation. These anatomical abnormalities affect pressure consonants and resonance balance, often resulting in impaired phoneme production and varying degrees of nasality. Understanding how CLP affects speech is essential for guiding rehabilitation and designing targeted early interventions.

This systematic review aimed to identify the most frequently affected speech phonemes and determine the degree of nasality in patients with CLP. A literature search covering the last 10 years (2015-2025) was conducted using PubMed, SciELO, and Scopus. A total of 484 articles were identified, of which 20 met the inclusion criteria. The most affected phonemes across languages were /k/, /p/, and /t/, all voiceless stop consonants. Most patients exhibited mild nasality; however, a consistent association was observed between delayed reconstructive surgery and increased nasality severity.

## Introduction and background

Cleft lip and palate (CLP) are a group of congenital malformations of the craniofacial complex. This problem is caused by an incomplete union of the facial processes during key periods of embryonic development [1].

Communication, seen from the neurological perspective, is one of the most complex activities that an individual develops together with society, since it is the coordinated activity of muscles and nervous mechanisms that result in the production of combined phonemes and the elaboration of sentences with syntax and grammar [2].

The daily lives of people with CLP will differ in many ways from those without this condition. Activities such as communicating, socializing, kissing, counting, speaking, smiling, and feeding themselves require additional effort [3].

According to the World Health Organization (WHO) [4], in 2021, between 1 and 1.5 per 1000 births resulted in a newborn with this pathology. According to Mena-Olalde et al. [5], Denmark has the highest reported incidence at 2.31:1000, followed by Tehran at 2.4:1000, Pakistan at 1.9:1000, Croatia at 1.71:1000, Ireland at 1.47:1000, Jordan at 1.39:1000, and Canada at 1.27:1000.

Navarrete et al. [6] indicate that the variability per 10,000 births in Spain is 3.12, while in Japan it is 20.97, 6.7 in New Zealand, and 13.35 in Norway, with China having the highest prevalence. In Latin America, in countries such as Colombia, the national study of oral health determined that 0.07% have CLP, followed by 0.04% with cleft lip only, and 0.02% with cleft palate only [7].

Epidemiological figures in Asian countries vary by region and methodology: China’s national analyses report overall orofacial cleft prevalence around 1.4 per 1,000 live births (≈14 per 10,000), with marked regional differences and some provinces reporting higher local rates [8]. South Korea has reported total orofacial cleft prevalences on the order of ~11 per 10,000 live births in population-based studies [9]. Studies and reviews covering multiple Asian countries show that prevalence estimates typically fall between ~1 and 2 per 1,000 live births (10-20 per 10,000), although values differ by country, region, and study design [9].

In Mexico, the national prevalence of cleft lip and CLP increased slightly from 2.4 and 2.5 per 10,000 births in 2008 to 3.0 and 3.0, respectively, in 2014 [6]. In our country, Ecuador, at the Pediatric Hospital "Baca Ortíz" in the period from January to December 2014, 196 patients with cleft lip and palate (FLAP) were analyzed. The prevalence was 66.8% among patients under three years of age and 33.2% among patients older than three years; as for the diagnosis, 27% had a unilateral right cleft lip, while 71% had a unilateral left cleft lip [10].

At the Isidro Ayora Hospital in Quito, Ecuador, 163 cases of malformations were reported between 2005 and 2010. Of these, 9.2% were cleft lip (15 cases), 23.9% were cleft palate (39 cases), and 66.9% were CLP (109 cases) [7].

Understanding the most affected phonemes and the degree of nasality present in people with CLP is essential for planning a practical therapeutic approach. Accurate identification of these articulatory and resonant alterations enables the design of early, targeted interventions to optimize speech production. Interdisciplinary work that integrates the evaluation and treatment of nasality and the affected phonemes favors more comprehensive and personalized care, significantly contributing to the well-being and quality of life of those with this condition.

This study aimed to determine which speech phonemes are most affected and to identify the degree of nasality in patients with CLP.

## Review

Methods

The present study was conducted based on a comprehensive bibliographic review of scientific databases, including articles relevant to CLP and their association with the phonetic function of the stomatognathic system. Information was systematically compiled from articles that met the predefined selection criteria and were identified in recognized scientific databases such as PubMed, SciELO, and Scopus, as well as through Google Scholar. Although Google Scholar is not a traditional scientific database but rather a broad academic search engine, it was included to ensure the retrieval of grey literature and potentially relevant studies not indexed in conventional databases, thereby enhancing the comprehensiveness of the search strategy.

The information collected was managed according to the Preferred Reporting Items for Systematic Reviews and Meta-Analyses (PRISMA) protocol [11], which facilitates systematic reviews and allows for the synthesis of the procedures used for data selection. In addition, the number of scientific articles identified, selected, chosen, and included in the study was specified (Figure 1).

**Figure 1:** PRISMA flow chart illustrating the study identification and selection process PRISMA: Preferred Reporting Items for Systematic Reviews and Meta-Analyses

The PICO question posed in this study was: In patients with cleft lip and palate, what are the most affected speech phonemes and the degree of nasality reported in the literature? P (Population): Individuals with cleft lip and palate; I (Intervention / Indicator): Assessment of articulatory performance and nasality; C (Comparison): Differences across languages, assessment methods, or surgical/therapeutic contexts (when applicable); O (Outcome): Identification of the phonemes most frequently affected and characterization of the degree of nasality.

Selection Criteria to Limit the Search

Articles published in the last 10 years (2015-2025), research related to CLP, studies on phonetic problems, articles in Spanish, English, and Portuguese, free full-text articles, randomized clinical trials and observational studies, and studies in people with CLP were included.

Search Strategy

The search strategy used to gather information for the study was through the use of MeSH/DeCS terms plus the combination of Boolean terms in the different databases, such as: "cleft lip" AND "phonetic", "cleft lip" AND "oral speech system", "Cleft lip" AND "Language and hearing sciences", "labio y paladar hendido" AND "habla", "cleft palate" AND "vocal rehabilitation", "cleft palate" AND "phonetic", "cleft palate" AND "speech system", "orofacial clefts" AND "phonemes"; "cleft palata" AND "nasality". 

Results

Seven studies focusing on children and adolescents with CLP are presented, in which speech articulation assessments were carried out. Difficulties in pronouncing certain phonemes were identified in all cases, varying according to the participants' language. In English, the most affected phonemes were /k/, /ʃ/, /p/, /t/, followed by /b/, /d/, and /g/. In Brazilian Portuguese, problematic phonemes included /k/, /b/, /d/, /g/, as well as /t/, /s/, and /z/. In Spanish, the consonants with the greatest difficulty were: /s/, /t/, /d/, /l/, /rr/, and /ll/. In Turkish, the most difficult phonemes were/p/, /t/, and /k/, while in Danish, difficulties were found with/k/, /f/, /p/, and /t/. Through analysis of all languages, it is observed that the most difficult phonemes, regardless of the language, are /k/, /p/, and /t/. These phonemes are classified as follows: /k/ is a voiceless velar stop consonant, /p/ is a voiceless bilabial stop, and /t/ is a voiceless dental stop (Table 1).

**Table 1:** Phonemes affected by cleft lip and palate according to language type

Author	Qualification	Population	Methodology	Results	Database	Country	Year
Cleland et al. [12]	An ultrasound investigation of tongue dorsum elevation in children with cleft palate +/- cleft lip	Recordings of 39 English-speaking children with cleft palate with or without cleft lip (CP/-CL) aged 3 to 12 years.	The speech materials include (1) counting from one to ten, (2) ten repetitions of all exercises with voiceless (or voiced if necessary) obstruents in the sequence /aCa/, (3) sentences from Great Ormond Street Speech Assessment 1998, (GOS.SP.ASS.'98),21, and (4) five pairs of minimal sets presenting common substitutions for the phonemes /s, ∫, t∫, t/ in various vowel contexts.	Typically developing children have higher dorsal excursion indices (DEIs) for /k/ and /ʃ/, and lower indices for /s/ and /t/. The difference in DEI between /k/ and /ʃ/ is smaller in children with CP+/-CL than in children with articulation disorders (AD).	Scopus	United Kingdom	2024
Hardin-Jones et al. [13]	Production of stop consonants in children with cleft palate after palatoplasty	Study participants included 113 English-speaking children with cleft palate ± repaired lip (mean age, 16 months) enrolled in the multicenter CORNET study.	Parents were asked to record approximately two hours of their children's vocalizations or words at home using a Language Environment Analysis recorder. Four 10-minute samples were extracted from each child's recordings to analyze the presence of oral stop consonants, with a minimum of 100 vocalizations required for analysis.	Preliminary results show that at least one oral stop was present in the consonant inventory of 95 of the 113 children (84%) at 16 months after surgery, and 80 of these children (71%) produced two or more different stop types. Approximately 50% of the children (57/113) made all three voiced stops, and eight children (7%) made all six stop consonants. 50% of the children had difficulty with voiced stop consonants such as /b/, /d/, and/g/, and 93% had trouble with voiceless stop consonants such as /p/, /t/, and/k/.	Scopus	USA	2024
Gölaç et al. [14]	Voice onset time (VOT) in Turkish-speaking children with repaired cleft lip and/or palate: a case-control study	Thirty-nine children with repaired cleft lip and/or palate (CL/P) and 39 healthy Turkish-speaking children were included in the study.	Clinical data such as age, sex, language spoken, hearing status, CL/P type, presence of lip/palate repair, results of speech and sound disorders examination, and presence of malocclusion and/or oronasal fistula were retrospectively collected. VOT values for the syllables /pa/, /ta/, and /ka/ were obtained using Praat software and compared between the study group (SG) and the control group (CG).	Voice onset time was slower in the study group for the syllables /pa/, /ta/, and /ká/, with p-values of 0.015, 0.045, and 0.037, respectively. Cleft lip and palate delay voice onset time.	Scopus	Türkiye	2024
Andrade et al. [15]	Influence of an Intensive Speech Therapy Program on the Speech of Individuals with Cleft Lip and Palate	Thirty-seven patients underwent surgery for cleft lip and/or palate; 16 women (43%) and 21 men (57%), all Portuguese speakers.	Voice recordings were obtained before and after the Intensive Speech Therapy Program (ISTP) in a sound-shielded environment using high-quality microphones. The recorded voice samples consisted of six sentences, each containing the six Brazilian Portuguese stop consonants (a total of 24 target consonants), distributed as follows: "p Papai olha a pipa.	The occlusive consonants that caused problems with glottal articulation were "k", "b", "d", and "g"; only "p" showed improvement. The articulation of the glottal stop was classified as present in 325 (37%) of the samples. Of those 325 (100%), 197 (61%) remained with this error, and 128 (39%) did not.	SciElo	Brazil	2023
Tenelanda et al. [16]	Speech problems associated with labial and palatal dysglossia	Forty-two patients using intentional nonprobability sampling, Spanish-speaking.	The study employed an observational technique, using dental clinical histories and a speech algorithm as tools. The clinical histories provided the medical-dental diagnosis, while the algorithm evaluated speech on a three-level scale using five indicators: nasolabial, elicited nasolabial, dentopalatine, velopharyngeal, and the stress test (blowing a balloon).	The most common is cleft palate with cleft lip, accounting for 59.6% of the study population. Most patients underwent surgery; these presented greater difficulty producing the dentopalatal phonemes /t/, /d/, /l/, /rr/, and /ll/. Twenty-five patients (59.5%) had a high level on the speech scale, and 17 (40.5%) had a medium level.	SciElo	Ecuador	2021
Jørgensen et al. [17]	Longitudinal study of the development of obstruent correction between three and five years of age in 108 Danish children with unilateral cleft lip and palate: a substudy within a multicenter randomized controlled trial	Audio and video recordings of 108/125 Danish participants aged 3 to 5, Danish speakers.	Audio and video recordings of a naming test were available for 108 children aged three and five years. Blinded raters phonetically transcribed the tapes. The naming test consisted of 24 words at age 3 and 27 words at age 5.	The phonemes most affected in Danish are /k/, /f/, /p/, and /t/. The phonemes that showed improvement were/ph, ts, kh/.	PubMed	Denmark	2020
Jacob et al. [18]	Oral diadochokinesia and lisp in speech production in children with surgically repaired cleft lip and palate	Thirty Portuguese-speaking children, aged 9 to 12 years, with complete unilateral cleft lip and palate and 30 with isolated cleft palate were studied.	Two speech-language pathologists evaluated repeated sentences containing the phonemes [s] and [z] to determine whether a lisp was present. Oral diadochokinetic ability was assessed by recording the rapid repetition of the syllables “ta” and “ka,” along with the sequence “pataka.” Inter-rater reliability was examined using the Kappa statistic. A Chi-square test was applied to compare the occurrence of lisping across the study groups, and independent t-tests were conducted to analyze diadochokinetic performance both between the groups and between participants with and without lisp.	In this sample, the phonemes most frequently impacted were /t/, /k/, /s/, and /z/. For the syllable “ta,” the mean diadochokinetic rates were 4.66 ± 0.61 repetitions per second in the cleft palate (CP) group and 4.65 ± 0.48 in the unilateral cleft lip and palate (UCLP) group, with scores ranging from 3.33 to 7.1. Regarding the syllable “ka,” the CP group obtained an average of 4.06 ± 0.46 and the UCLP group 3.86 ± 0.58, within a range of 3.18 to 6.6. For the tri-syllabic sequence “pataka,” the results were 1.64 ± 0.16 for the CP group and 1.67 ± 0.16 for the UCLP group.	SciElo	Brazil	2015

Table 2 includes 13 studies on children with CLP, spanning an age range of 3 to 12 years. The most studied age group was 6 to 12 years (8/13 articles). All studies were conducted in patients with CLP; however, the majority (6/13) focused on unilateral clefts, while a few articles (2/13) addressed bilateral clefts. All individuals underwent corrective surgery before evaluation of nasality. Most articles (9/13) indicated that the subjects underwent primary surgery, with the most frequently mentioned techniques being primary palatoplasty (4/9 articles), two types of flaps (2/9 articles), vomer flap (1/9 articles), and pharyngeal flap (1/9 articles). Additionally, some articles (2/9) mentioned primary repair without specifying the technique; on the other hand, a small number of studies (4/13) did not clarify either the type or the repair technique. All studies included tests to assess nasality in patients with CLP. Most studies (7/13) classified nasality as mild, moderate, and severe, with averages of 55.53%, 19.38%, and 9.57%, respectively. Few studies (4/13) reported nasality, with an average of 57%. Finally, the minority of articles (2/13) compared nasality based on two groups: early and late repair. These studies found that, as reconstructive intervention was delayed, the severity of nasality increased. In this regard, mild nasality was observed in 34.65% of patients who underwent early surgery, compared with 21.85% of those who underwent later surgery. Moderate nasality was observed in 30.8% of cases with early intervention, compared to 32.25% of those with delayed surgery. Finally, severe nasality was observed in 32.90% of patients with early intervention, compared to 38.5% of those with delayed surgery. To facilitate a clearer understanding of the results, Table 3 summarizes the information presented above.

**Table 2:** Degree of nasality in patients with cleft lip and palate

Author	Qualification	Population	Methodology	Results	Database	Country	Year
Okhiria et al. [19]	Longitudinal data on speech outcomes in internationally adopted children compared with non-adopted children with cleft lip and palate	Twenty-three adopted international (AI) children from China were matched with 23 non-adopted (NA) children born in Sweden.	Experienced speech-language therapists blindly re-evaluated audio recordings from routine follow-ups at ages 5 and 10 years. Velopharyngeal function (VPF) was assessed with the Velopharyngeal Competence Composite Score (VPC-Sum) for individual words and rated on a three-point scale administered by Uppsala University, Velopharyngeal Competence Rating (VPC-Rate) for sentence repetition.	Fifty percent of children presented hypernasality at age 5, while 93% at age 10. For the second evaluator, 79% of patients showed nasality at age 5, while 64% showed it at age 10. Finally, for the third evaluator, 71% presented hypernasality at age 5, and 93% at age 10.	Scopus	China	2023
Malmenholt et al. [20]	Speech feature profiles in five-year-old Swedish children with speech sound disorders related to suspected childhood apraxia of speech or cleft palate	34 participants	All participants underwent assessment using the standardized SVANTE instrument. The task involved naming 74 picture stimuli designed to prompt single-word productions. Of these, 49 were monosyllabic items featuring different consonant–vowel patterns (including CV, CVC, CVCC, CCV, CCVC, VC, and VCV structures), and 25 were disyllabic items incorporating patterns such as VCCV, VCVC, CVCV, CVCVC, CCVCV, and CCVCVC. Testing took place in a quiet environment, and speech samples were captured via video and/or audio using a digital recording device. For notation, C represents a consonant and V represents a vowel.	76% of the population had hypernasal resonance, and 88% had consonant distortion.	Scopus	Sweden	2022
Rezaei et al. [21]	Speech outcomes after palatal closure in children of seven years	One hundred and eighty clinical records were collected. This population included 102 boys (56.7%) and 78 girls (43.3%). The mean age at palatal surgery and speech evaluation was 16.7 ± 11.97 months (range: 5 to 72 months) and 53.47 ± 15.18 months (range: 36 to 84 months), respectively.	The medical records of 180 preschool-aged children with repaired cleft palates were reviewed. The percentage of children with hypernasality, nasal emission, nasal turbulence, and compensatory disarticulations was calculated. The relationship between cleft type and age at the time of palatal surgery, as independent variables, and speech outcomes was examined.	The early-surgery group showed hypernasality in 82.6% of cases. Of these, 20.9% were mild, 19.7% moderate, and 41.9% severe. The late surgery group presented hypersensitivity in 85.2% of cases, with mild in 11.1%, moderate in 21%, and severe in 53.1%.	Scopus	Iran	2022
Koh et al. [22]	Speech outcomes in five-year-old Korean children with bilateral cleft lip and palate	A retrospective study was conducted in 52 children with complete BCLP who underwent primary palatal surgery at a tertiary medical center. 44 boys and 8 girls.	All participants underwent their routine speech evaluations at the age of five. These follow-up assessments were administered and recorded by one of two speech-language pathologists affiliated with the clinic. The recorded material included standardized speech tasks such as word lists from the Standardized Articulation Test and the Ural Test of Articulation and Phonation, numerical counting from one to ten, and repetition of sentences emphasizing different vowel heights (high, low, and mixed).	63.5% of participants showed evidence of hypernasality ranging from normal to mild. 15.4% presented mild to moderate hypernasality. The results also revealed that 21.2% of participants showed a moderate or higher degree of hypernasality that clearly required clinical management: 15.4% had moderate, 3.8% moderate to severe, and 1.9% severe.	Scopus	Korea	2022
Fitzpatrick et al. [23]	The impact of hearing loss on speech outcomes in five-year-old children with cleft palate ± cleft lip: a longitudinal cohort study	Eighty-five children with the Cohen method	A spontaneous speech sample was collected, counting from one to 20 and from 60 to 70, respectively, and a nursery rhyme and phrases taken from the Great Ormond Street speech assessment were recited and video-recorded. A consensual listening process was used by two cleft specialists, speech-language therapists (SLTs), who listened to the recordings and classified the children's speech.	Eighty-nine percent had a green (dark or light) nasality result. An amber or red nasality result was found in 3% of the sample. Developmental errors were present in 57% of children, and 3% had missing data.	Scopus	United Kingdom	2021
Safarpour et al. [24]	Analysis of language samples in children with cleft lip and palate	Fifty-eight Persian-speaking children (28 children with cleft lip and palate (CLP) and 30 children without craniofacial anomalies = no clefts).	The children's language samples were collected using the picture description method. The children's 50 consecutive intelligible utterances were analyzed using the Persian Developmental Sentence Scoring (PDSS) as a clinical morpho-syntactic measurement tool.	The majority of children studied (92%) were diagnosed with mild to severe hypernasality and nasal air emission.	Scopus	Iran	2021
Bettens et al. [25]	Speech perceptual outcomes after early primary palatal repair in Ugandan patients with cleft palate	Twenty-four Ugandan children	Three speech-language pathologists (SLPs) with professional experience ranging from three to eight years independently carried out the perceptual evaluations of cleft speech characteristics (CSC). Two evaluators had specific training in applying the Cleft Audit Protocol for Speech–Augmented (CAPS-A). The recorded speech samples were presented in random order and assessed using standard on-ear headphones.	71% of the patients were judged to have normal resonance or borderline hypernasality, and 29% had mild to moderate hypernasality. In contrast, none of the children in the control group had these articulation errors.	Scopus	Uganda	2021
Boyce et al. [26]	Exploring speech and language in individuals with non-syndromic submucous cleft palate: a preliminary report	Fifteen participants with submucous cleft palate (SMCP) aged five years	Speech and resonance were evaluated following a standardized cleft speech assessment procedure. This protocol included automatic speech tasks such as counting, a spontaneous conversational sample, and a set of sentences designed to test all English consonants and clusters in various word positions. Speech intelligibility was scored on a four-point scale, where 0 indicated completely clear speech and 3 denoted severely reduced intelligibility.	2 of 15 patients had mild hypernasal resonance, and 3 had accompanying nasal air emission or turbulence.	Scopus	Australia	2019
Zulkipli et al. [27]	A perceptual assessment of resonance disorders in children with unilateral cleft lip and palate repair at Universiti Sains Malaysia Hospital	Four children with cleft lip and palate (CPLP) repaired at USM Hospital, aged between 8 and 12 years, were included.	After the participants' speeches, samples were collected. Conversational speech was first collected by establishing rapport with the participants. Participants were then asked to read a series of speech stimuli in Bahasa Melayu, and their speech samples were recorded using an audio recorder and used for data analysis for the study.	75% (3/4) of participants exhibited hypernasality as the type of resonance disorder, and 25% (1/4) had no evidence of hypernasality or any other kind of resonance disorder.	Scopus	Malaysia	2018
Safaiean et al. [28]	Speech intelligibility after cleft lip and palate repair	Seventy-four monolingual Persian-speaking children, 32 children with repaired Cleft Lip and Palate (CL/P), and 32 controls aged 3–5 years	Speech intelligibility was assessed using the Persian Speech Intelligibility Test, which was normed in children aged 3 to 5 years. Each speech sample was listened to by a speech-language pathologist (SLP) and two lay speech therapists. Two objective measures of speech intelligibility were used in this study, including the Percentage of Correct Consonants (PCC) and the Percentage of Wise Words (PIW).	Nearly 90% of children with Cleft Lip and Palate (CL/P) presented with mild to severe hypernasality (mild = 34.4%, moderate = 34.4%, and severe = 21.9%). The results revealed a significant relationship between hypernasality severity and speech intelligibility in children with CL/P.	Scopus	Iran	2017
Menegueti et al. [29]	Speech profile of patients undergoing primary palatoplasty	Ninety-seven patients of both sexes with cleft palate and/or cleft and labial palate participated.	Auditory-perceptual speech evaluation. A specific protocol developed by the Clinic is used for these evaluations. It was prepared by the speech-language pathology (SLP) Clinic following an extensive literature review and participation in thematic meetings to standardize evaluation protocols for patients with cleft palate. This protocol includes an evaluation of the mouth's morphology, the motor system, occlusal function, and speech.	Hypernasality was present in 72.1% of the early intervention group and 85.2% of the late intervention group. Hypernasality was absent in 27.9% of the early intervention group and 14.8% of the late intervention group.	SciElo	Brazil	2017
Sell et al. [30]	Study on cleft care in the United Kingdom (UK) Part 4: Speech perceptual outcomes	Two-hundred and forty-eight children were born with a complete unilateral cleft lip and palate	Specialized speech and language therapists (SLTs) at the center recorded speech audio and video according to nationally agreed guidelines. Two independent listeners performed perceptual analysis using the Cleft Audit Protocol for Speech–Augmented (CAPS-A) audit tool. These findings suggest that centralizing cleft care in high-volume centers has improved speech outcomes in the Kingdom.	Children from Cleft Care UK (CCUK) presented 10.2% hypernasality, while children from Clinical Standards Advisory Group (CSAG) presented 17.6%	Scopus	United Kingdom	2015
Ganesh et al. [31]	A randomized controlled trial comparing two techniques for unilateral cleft lip and palate: growth and speech outcomes during the mixed dentition	Eighty-five patients (40 patients in the vomer flap (VF) technique group and 45 patients in the two-flap (TF) technique group). These patients were in the age range of 7 to 9 years,	Two speech-language pathologists, experienced in cleft lip and palate, independently assessed the speech samples. The speech samples were blinded and randomized before the perceptual assessment. For the perceptual evaluation, universal parameters were used to report the results.	In the VF group, 17.6% had moderate hypernasality. In the TF group, 2.6% had moderate hypernasality.	PubMed	India	2015

**Table 3:** Interpretative summary of speech phonemes and nasality results

Category	Findings
Age range	3–12 years
Most studied age group	6–12 years (8/13 studies)
Type of cleft	All cleft lip and palate; unilateral (6/13), bilateral (2/13)
Surgical status	All participants underwent corrective surgery before nasality assessment
Primary surgery details	Reported in 9/13 studies
Surgical techniques	Primary palatoplasty (4/9), two-flap palatoplasty (2/9), vomer flap (1/9), pharyngeal flap (1/9), unspecified primary repair (2/9)
Studies not reporting technique	4/13
Nasality assessment	All studies included nasality testing
Nasality classification (7/13 studies)	Mild: 55.53%; Moderate: 19.38%; Severe: 9.57%
Studies reporting only “nasality present”	4/13 studies (average: 57%)
Studies comparing early vs. late repair	2/13
Nasality by timing of surgery	Early repair: Mild 34.65%, Moderate 30.8%, Severe 32.9% Late repair: Mild 21.85%, Moderate 32.25%, Severe 38.5%
Conclusion from timing comparison	Delayed surgery increases nasality severity

Discussion

This research established that individuals with CLP experience difficulties with phonetic articulation due to the nature of their condition, which involves a lack of continuity between hard and soft tissues during fetal development. The research revealed that the affected phonemes vary depending on the language spoken by the individual; however, the most common, regardless of language, are /k/, /p/, and /t/. Similar results are reported by Moreno and Sarmiento [32], who, upon reviewing the medical records of children with this condition, concluded that the most affected phonemes are those under high pressure, such as /t/ and /s/. Along the same lines, Matos [33] also observed that, in Spanish, the phonemes with articulation problems were /b/, /d/, /s/, /p/, and /k/. Rodríguez [34] added that, due to poor control of aspirated air when speaking, errors occurred in occlusive phonemes such as /p/, /t/, and /c/. Consistent with these findings, Pandit et al. [35] reported that the velar sound group presented the highest number of errors, followed by the palatal, dental, and labial groups. Similarly, Southby et al. [36] mentioned that participants with cleft palate showed posterior articulation errors in phonemes such as /k/. However, some results contradict the data of this thesis. Similarly, Tenelanda et al. [37] noted that the phonemes /k/, /g/, /j/, /x/, /c/, /ch/, /ñ/, /ll/, and /y/ tend to pose greater communication difficulties. Likewise, Shin and Kim [38], when evaluating two patients, found that most of the errors were distortions secondary to nasalization, as in the case of /s'/ and /t'/. On the other hand, Finnegan [39] highlighted that the contrasts of the following phonemes /p/-/b/, /ʃ/-/ʒ/, and /tʃ/-/dz/ constituted 60.5% of all voicing errors in the CLP group.

This research revealed that most patients presented a mild degree of nasality, which was lower when the intervention was performed at an early age. Ooppanasak et al. [40] found that, when comparing speech characteristics of children with CLP with those of children without pathology, 66% of children undergoing cleft repair showed a degree of nasality ranging from mild to moderate. Van Lierde et al. [41] reported that 49% of those evaluated perceived their nasality as mild and recommended speech therapy to reduce this perception further. Likewise, Chwa et al. [42] concluded that patients who presented a higher degree of nasality (hypernasality) were those treated late, that is, after 18 months. This phenomenon is common in developing countries, including those in Central and South America and Africa. Along the same lines, Ozgur et al. [43] reported that, in their comparative study of surgical protocols, the group that received traditional palatoplasty at an early age showed mild nasality. In contrast, those who underwent radical intravelar veloplasty showed moderate nasality.

Reported degrees of nasality after primary palatal repair vary across cohorts and assessment methods, but several consistent patterns emerge. Some studies report a large proportion of children with only mild or no hypernasality when surgery and multidisciplinary care are performed early and when postoperative speech therapy is available, while other series, especially those from settings with delayed repair, report high rates of moderate/severe hypernasality. For example, Larangeira et al. [44] found important differences in nasality results depending on the evaluation method used (live perceptual judgement, recorded samples, nasometry), underlining that the measurement technique affects the reported prevalence of nasality. Rezaei et al. [20] reported that 67.7% of their preschool cohort demonstrated moderate or severe hypernasality and that later age at palatoplasty was significantly associated with both compensatory misarticulations and higher degrees of hypernasality. 

Where included studies report the proportion with mild nasality specifically, the values are heterogeneous and depend on population, surgical protocol, and assessment method. Some perceptual studies report that roughly half of evaluated children are judged to have mild nasality or better, whereas other series, particularly those with late repairs, show a majority with moderate/severe nasality. These discrepancies stress that a single pooled percentage for “mild nasality” is not robust without harmonized assessment methods and comparable patient populations [45].

On the other hand, Sireesha et al. [46] noted that although surgical interventions aim to eliminate clefts and reduce hypernasality, this characteristic may persist in individuals regardless of the age of intervention. In contrast, the study by Hashemi et al. [47] found that among 100 school-aged children with CLP who received speech therapy and underwent early surgery, those with additional syndromes were 6 times more likely to exhibit a higher degree of hypernasality than those without associated conditions. However, nasality at mild levels was observed in all cases.

## Conclusions

In conclusion, the present study identified the most difficult phonemes to articulate across languages (English, Portuguese, Spanish, and Turkish) as /p/ (voiceless bilabial), /k/ (voiceless velar), and /t/ (voiceless dental). All patients had undergone primary palatoplasty, with no specification of the protocol or surgical technique used. Regarding speech resonance, the majority presented mild nasality, while moderate nasality and severe nasality were less common. However, a worrying trend was evident: delay in reconstructive surgery was associated with an increase in the severity of nasality.
